# Bone regenerative medicine: classic options, novel strategies, and future directions

**DOI:** 10.1186/1749-799X-9-18

**Published:** 2014-03-17

**Authors:** Ahmad Oryan, Soodeh Alidadi, Ali Moshiri, Nicola Maffulli

**Affiliations:** 1 Department of Pathology, School of Veterinary Medicine, Shiraz University, Shiraz 71345, Iran; 2 Division of Surgery and Radiology, Department of Clinical Sciences, School of Veterinary Medicine, Shiraz University, Shiraz 71345, Iran; 3 Department of Tissue Engineering and Regenerative Medicine, Reproductive Biotechnology Research Center, Avicenna Research Institute, ACECR, Tehran 3197619751, Iran; 4 Department of Musculoskeletal Disorders, School of Medicine and Surgery, University of Salerno, Salerno 84084, Italy; 5 Centre for Sports and Exercise Medicine, Queen Mary University of London, Barts and the London School of Medicine and Dentistry, Mile End Hospital, 275 Bancroft Road, London E1 4DG, UK

**Keywords:** Bone graft, Tissue engineering, Regenerative medicine, Three-dimensional printing, Orthopedic research

## Abstract

This review analyzes the literature of bone grafts and introduces tissue engineering as a strategy in this field of orthopedic surgery. We evaluated articles concerning bone grafts; analyzed characteristics, advantages, and limitations of the grafts; and provided explanations about bone-tissue engineering technologies. Many bone grafting materials are available to enhance bone healing and regeneration, from bone autografts to graft substitutes; they can be used alone or in combination. Autografts are the gold standard for this purpose, since they provide osteogenic cells, osteoinductive growth factors, and an osteoconductive scaffold, all essential for new bone growth. Autografts carry the limitations of morbidity at the harvesting site and limited availability. Allografts and xenografts carry the risk of disease transmission and rejection. Tissue engineering is a new and developing option that had been introduced to reduce limitations of bone grafts and improve the healing processes of the bone fractures and defects. The combined use of scaffolds, healing promoting factors, together with gene therapy, and, more recently, three-dimensional printing of tissue-engineered constructs may open new insights in the near future.

## Introduction

Unlike other tissues, the bone can regenerate and repair itself: in many instances, bone injuries and fractures heal without scar formation [1,2]. Nevertheless, in pathological fractures or large and massive bone defects, bone healing and repair fail. Insufficient blood supply, infection of the bone or the surrounding tissues, and systemic diseases can negatively influence bone healing, resulting in delayed unions or non-unions [3-6]. Bone is the second most commonly transplanted tissue after blood [2,7]. A bone graft is defined as an implanted material that promotes bone healing alone or in combination with other material(s) [7], through osteogenesis, osteoinduction, and osteoconduction [8], in combination or alone.

The selection of an ideal bone graft relies on several factors such as tissue viability, defect size, graft size, shape and volume, biomechanical characteristics, graft handling, cost, ethical issues, biological characteristics, and associated complications [9]. The materials used in bone grafting can be divided into several major categories, including autografts, allografts, and xenografts. Synthetic and biologically based, tissue-engineered biomaterials and combinations of these substitutes are other options [10]. Each of these options has advantages and disadvantages. Allografts and xenografts have osteoinductive and osteoconductive characteristics but lack the osteogenic properties of autografts [9-11]. Autografts are the ‘gold standard’ in reconstructing small bone defects and have strong osteogenic characteristics relevant to bone healing, modeling, and remodeling [12]. Pain and donor site morbidity as well as other risks such as major vessel or visceral injuries during harvesting are some of the disadvantages of autografts [13]. For these reasons, several alternative options have been introduced and tested [14,15]. Allografts are an alternative option with major limitations associated with rejection, transmission of diseases, and cost. Allografts have lower incorporating properties with the host healing tissues as compared with autografts [13,16,17]. Xenografts, in addition to the disadvantages of allografts, carry the risks of transmission of zoonotic diseases, and rejection of the graft is more likely and aggressive [17,18]. Given these problems, tissue engineering has been introduced in the last decade. Tissue engineering involves using relevant scaffolds, introducing appropriate growth factors and cells, and, more recently, the use of stem cells [17]. Using tissue engineering techniques, it is possible to design new scaffolds and tissue grafts aiming to decrease the disadvantages of traditional grafts and improve graft incorporation, osteogenicity, osteoconductivity, and osteoinductivity [10,17].

Tissue engineering has limitations, including use of a wide variety of materials in producing tissue-engineered grafts or scaffolds. Consequently, translational investigations testing each material are limited, reducing their clinical applicability. Therefore, some important aspects of host graft interaction and immune response to these implants, scaffolds, and viable grafts are still not clear [17]. With advances of tissue engineering, the ability to repair or regenerate bone tissue is developing, and its applications are expanding. In this review, we discuss some of the available scientific evidence on different types of bone graft, their characteristics, and their advantages and disadvantages. Moreover, we highlight the application of tissue engineering techniques to overcome the limitations of the available grafts and to improve bone regeneration.

## Structure and properties of grafts and bone substitutes

### Structure of bone grafts

The cortical bone has higher mineral contents than the trabecular or cancellous bone [9]. In addition, given the presence of spaces within the structure of cancellous bone, the latter is more osteogenic than cortical bone [2]. The compressive stiffness and strength of the cortical bone are much higher than those of the cancellous bone. In selecting a graft or combination of grafts, the surgeon must be aware of these fundamental differences in bony structures [2,7]. Bone grafts may be cortical, cancellous, or cortico-cancellous (scanning ultramicrographs of different bone grafts are presented in Figure 1) [2].

**Figure 1:** **SEM ultramicrographs of microstructure of natural bone grafts. (A)** Trabecular or cancellous bone graft. Note the porous honey comb-like microstructure of cancellous bone graft. **(B)** Cortico-cancellous bone graft. **(C)** Cortical or compact bone graft (scalebars **(A-C)** 100 μm).

Cortical bone grafts are used mostly for structural support and strength, and cancellous bone grafts for osteogenesis. Structural support and osteogenesis may be combined, one of the most important advantages of using cortico-cancellous bone grafts [9]. Cancellous bone grafts are commonly used in fracture non-union, dental defects, maxillofacial defects, spinal fusion, and other small bone defects [19,20]. These grafts lack mechanical strength, but are easy to use. The porous structure of cancellous bone grafts can enhance bony ingrowth and improve healing, allowing faster revascularization [19].

Cortical bone grafts are applied less frequently, and they may be used as onlay grafts [21]. Onlay bone graft is used to augment atrophic bone outside the anatomical boundaries of the skeleton. An example of an onlay graft is the graft needed to increase the atrophic alveolar bone width of a future implant site. This three-dimensional positioning of the graft has a major role on the course of healing and thus on the graft success and outcome of incorporation [7]. When a graft is used to fill a bone defect within the confines of the anatomical skeleton, the term inlay graft is more appropriate [16]. Onlay grafts undergo a more complicated healing course than inlay grafts [7].

The resorption rate of the onlay grafts is higher than the inlay grafts for two reasons: (1) the onlay grafts are less exposed to the recipient bone vasculature, which results in decreased bone remodeling; (2) the onlay bone grafts are exposed to forces from the surrounding soft tissues leading to more osteoclastic resorption in the areas exposed to these forces [7,16].

### Properties of bone grafts

To decide which graft is more appropriate for a given condition, understanding of the biological properties of each graft is necessary. An ideal bone graft material should have osteogenesis, osteoinductivity, osteoconductivity, and osseointegration characteristics [2,8,22].

Osteogenesis is the capacity to produce new bone by the osteoblasts by differentiation of osteoprogenitor cells either present in the recipient bone or coming from the graft material. This property is mainly present in autogenous grafts as compared with allografts and xenografts, because the cellular structures of the allografts and xenografts have low viability after implantation [23,24].

Osteoinduction is the capability of the graft materials to induce formation of the bone-forming cells via differentiation of multipotent mesenchymal stem cells (MSCs) of the surrounding host tissues to produce osteoprogenitor cells followed by development of osteoblasts. Such ability has been discovered in growth factors including bone morphogenetic proteins (BMPs) such as BMP-2 and BMP-7, transforming growth factor-β (TGF-β), fibroblast growth factor (FGF), insulin-like growth factor (IGF), and platelet-derived growth factor (PDGF) [2,8,22,24,25].

Osteoconduction is a characteristic whereby the graft acts as a permanent and resorbable scaffold, mechanically supporting ingrowth of vessels and new bone from the borders of the defect into and onto its surfaces. This characteristic initiates or induces new bone formation [8,22,24,25]. Finally, osseointegration is the ability to bind to the surrounding bone without an intervening layer of fibrous tissue, allowing incorporation of the graft at the host site [8]. All bone grafts and bone-graft substitute materials can be described by these processes [23].

Among all types of bone grafts, only autografts possess all the above features. Allografts and xenografts exhibit only two or three of the four features of an ideal bone graft material (osseointegration, osteoconduction, and perhaps osteoinduction) and lack osteogenic properties [6,8].

### Incorporation of bone grafts

Incorporation of bone grafts within the recipient bone bed depends on factors such as graft revascularization. Fast incorporation and suitable healing of the graft can be obtained with optimal quality and speed of revascularization if there is adequate independent vascular supply to the defect site [7,13]. In non-vascularized grafts, the blood vessels slowly penetrate from the recipient bone into the graft, and the healing time is thus prolonged [16,26]. Incorporation of each graft depends on these properties, which can vary based on the source (auto-, allo-, or xenograft), and structure of the graft (cancellous or cortical bone) [13,16].

Regardless of the source or structure, all transplanted bone grafts proceed through five stages: inflammation, revascularization (capillary buds invade the graft), osteoinduction (differentiation of multipotent cells into osteoblasts), osteoconduction (ingrowth into the graft by means of the host), and finally remodeling [13,21]. The duration of each phase can vary depending on the characteristics of the graft. Interference with vascularization, including infections and excessive micromotion at the reconstructed area, will delay incorporation [7,16]. For cortical grafts, vascularization is slower and occurs along Haversian canals, while it is performed by creeping substitution in cancellous grafts [13,16]. In the latter process, the newly formed osteoblasts line the trabeculae to form new bone simultaneous to resorption of bone by osteoclasts; while in cortical bone grafts, osteoclastic resorption is a prerequisite before osteoblasts can produce new bone. In other words, from the perspective of incorporation, the major difference between the cancellous and cortical autografts is that bone resorption precedes bone formation in the latter [13,16].

During the second and third stages, the immune system of the recipient becomes sensitive to the donor antigenicity [21]. Incorporation of cancellous autografts is fastest and most complete, followed by cortical autografts, cancellous and cortical allografts, and xenografts, respectively. Because allografts and xenografts are not genetically matched, they can initiate an immune response in the recipient. When allografts and xenografts are used, therefore, it is more likely that the graft will fail and the donor tissue is rejected [13,16,21]. Fresh allografts and xenografts produce stronger immunologic responses than fresh-frozen or freeze-dried allografts and xenografts [27].

### Immune response against bone grafts and substitutes

Th1 lymphocytes produce pro-inflammatory cytokines such as interleukin-2 (IL-2), interferon- γ (IFN-γ), and tumor necrosis factor-β (TNF-β) leading to macrophage activation, and can be associated with poor tissue remodeling and rejection of both allo- and xenograft transplants [28,29]. On the other hand, Th2 lymphocytes produce IL-4, IL-5, IL-6, and IL-10 cytokines that do not activate macrophages and are probably associated with graft incorporation [28,29].

Macrophages are characterized as M1 or M2 based on receptor expression, function, and production of cytokines [30]. M1 macrophages produce large amounts of pro-inflammatory cytokines such as IL-12 and TNF-α, which promote inflammation and express CD68 and CD80 surface markers in rats. On the other hand, M2 macrophages produce large amounts of IL-10 and TGF-β, inhibit the release of pro-inflammatory cytokines, promote constructive tissue remodeling, and express CD163 surface markers in rats [30,31]. M2 macrophages induce the Th2 lymphocyte response which is beneficial for tissue remodeling [30]. The presence of cellular material within extracellular matrix (ECM) of scaffold modulates the phenotype of the macrophages and lymphocytes involved in the recipient immunity response after implantation; this can be related to tissue remodeling outcome in terms of acceptance or rejection [30,31]. Indeed, a cellular graft elicits M1 macrophage and Th1 lymphocyte response and can result in the deposition of connective tissue and rejection of the graft. An acellular graft elicits M2 macrophage and Th2 lymphocyte response, leading to more constructive tissue remodeling outcome and acceptance of the graft [30].

### Types of bone grafts

Auto-, allo-, and xenografts as well as bone graft substitutes are all used to improve and enhance healing of bone defects (Figure 2). Autografts have limitations in pathologic fractures and massive bone defects; therefore, other types of grafts have been introduced to overcome the limitations of autografts in such situations [2,10,13]. All the available and alternative options have limitations and merits (Table 1), and selection of a proper graft or combination of them depends on the surgeon's preference and experience.

**Figure 2:** **Types of bone grafts. (A)** Autograft: The surgeon harvests bone from another site of the patient's skeleton, often from the iliac crest, and implants it into the bone defect site. This type of bone grafts leads to two surgeries, thus, two scars, more pain, and additional infection risk. **(B, C)** Allograft and xenograft: Here the bone graft is obtained from a human donor or animal model, respectively. These types of bone grafts, particularly xenografts, carry the risk of immunologic response and transmission of viral and bacterial disease and with xenografts, zoonotic disease. **(D)** Synthetic bone graft substitute: There are different types of synthetic grafts. These biomaterials are safe and need no second surgery site.

**Table 1:** Some advantages and disadvantages of the most commonly used three types of bone grafts

**Bone graft**	**Advantages**	**Disadvantages**
Autografts	Optimal osteogenic, osteoinductive, and osteoconductive properties; gold standard for bone grafting; without the risks of immunogenicity and disease transmission	Pain and morbidity in the donor site, limited quantity and availability, need for further surgery, hematoma, infection, the need for general sedation or anesthesia, longer operative time, and blood loss
Allografts	Osteoinductive and osteoconductive properties, without donor site morbidity, possible with local anesthesia, high availability, easy handling	Lack of osteogenic properties, potential antigenic response and disease transmission, variable osteoinductivity, limited supply, loss of biologic and mechanical properties due to its processing, non-availability worldwide due to religious and financial concerns and increased cost
Xenografts	Osteoinductive and osteoconductive properties, low cost, high availability	Lack of osteogenic properties, the risk of immunogenicity and transmission of infectious and zoonotic diseases, poor outcome

### Autografts

Bone grafts that are harvested from one site and implanted into another site within the same individual are termed autografts, autologous, or autogenous bone grafts [32]. They may be cancellous or cortical (non-vascularized or vascularized) bone, and in some instances a combination of both, ‘cortico-cancellous grafts’ [2,33]. Fresh autografts contain surviving cells and osteoinductive proteins such as BMP-2, BMP-7, FGF, IGF, and PDGF [9,22]. From a biological point of view, they are the best material available, since they totally lack immunogenicity. They retain their viability immediately after transplantation, and the lack of immunogenicity enhances the chances of graft incorporation into the host site [34]. Furthermore, the osteogenic, osteoinductive, and osteoconductive properties of fresh autografts are optimal, given the presence of MSCs, osteoprogenitor cells, osteogenic cells, and growth factors [24,35]. Autografts have no associated risk of viral transmission; moreover, they offer structural support to implanted devices and, ultimately, become mechanically efficient structures as they are incorporated into the surrounding bone through creeping substitution [23]. The main drawback is that autografts must be harvested from another body site, which implies additional surgery with a higher chance of donor site pain, morbidity, and complications [34]. If massive grafting is needed, adequate amounts of autograft may not be available, and other bone graft materials have to be considered [18,21].

Various sites have been used for harvesting the grafts' tissues. Grafts can be obtained from the iliac wing or crest, the proximal or distal tibia and radius, the proximal humerus, the distal ulna, ribs, calcaneus, and the proximal olecranon [36-41]. These sources each have advantages and disadvantages (Table 2). Among them, the iliac crest has notable advantages, such as easy access and availability of sufficient amounts of both cortical and cancellous bones [37,38,42]. Nevertheless, graft harvesting from this site can produce nerve, arterial, and urethral injury; pelvic fracture; and pain at the donor site [37,41]. Therefore, other sites such as the distal radius have been used [43,44]. Kitzinger et al. [44] compared the iliac crest and distal radius as the sources of bone graft in 18 patients; the distal radius can be a more suitable alternative, as, in their setting, it obviated the need for general anesthesia, reduced the duration of the operation, and involved a smaller surgical exposure. The greatest chance for successful transplantation of live bone is associated with a cancellous autograft or pedicled, vascularized cortical autograft [16,26]. In general, the success of grafting the autogenic bone depends on the survival and proliferation of the osteogenic cells, conditions at the recipient bed, type of graft chosen, handling of the graft, and shaping of the graft during the operative procedure to adapt it into the host's bone [39]. While fresh autologous graft has the capability of supporting new bone growth by all four means (induction, genesis, conduction, and integration), it may not be necessary for a bone graft replacement to inherently have all four properties in order to be clinically effective. When inductive molecules are locally delivered on a scaffold, the mesenchymal stem cells are ultimately attracted to the site and are capable of reproducibly inducing new bone formation, provided that minimal concentration and dose thresholds are met [23].

**Table 2:** Advantages and disadvantages of some sources of harvesting bone grafts

**Source**	**Advantages**	**Disadvantages**
Iliac crest	Large bone volume, rich source of progenitor cells and growth factors, easy access, providing both cancellous and cortical bones	Nerve, arterial, and urethral injury, increased blood loss, hematoma, infection, chronic post-operative donor site pain, high patient morbidity, high recovery time, large scar, hip subluxation, pelvic fractures, costly, local infection
Distal radius	Lower bone turn-over than iliac crest, lower post-operative pain than the iliac crest, easy to harvest, small incision is needed	Superficial radial nerve injury, fracture, infection
Tibia	Easy to access, less operative time, and less gait disturbance than the iliac crest	Fracture, less bone volume than iliac crest, infection

### Allografts

Allografts are harvested from one individual and implanted into another individual of the same species [13]. Given the limitations associated with harvesting autografts, allografts have been applied clinically and experimentally as a common alternative to autografts [45]. Bone allografts are distributed through regional tissue banks and by most major orthopedic and spinal companies [23].

Allografts are used in both morselized and structural forms [24] and are provided as cortical, cancellous, or cortico-cancellous grafts [22] and in various shapes such as powder, cortical chips, and cancellous cubes. They also can be processed as mineralized or demineralized, fresh, fresh-frozen, or freeze-dried forms [27,32]. Allografts can be obtained from cadavers or living donors. The cadaveric form is available as a commercial product [32]. Allografts obtained from fresh cadavers with preservation of their cellular and organic content are minimally processed [27]. The major advantages of allografts are their ready availability in various shapes and sizes, avoidance of the need to sacrifice host tissues, and no challenges of donor site morbidity [21,23]. Allografts have variable osteoinductive and osteoconductive properties but lack viable cells and, therefore, have lower osteogenic potential than autografts [32].

Bone allografts carry the risk of transmitting bacterial contamination and viral diseases, such as HIV and hepatitis B and C, and also they may induce immunological reactions that interfere with the bone healing process and can lead to rejection of the graft [17,18,21,22]. In addition, the rate of healing, using allografts, is generally lower than the autografts.

Given the higher chance of immune response initiation and the risk of disease transmission, fresh bone allografts are seldom used. With frozen and freeze-dried allografts, these concerns are partly obviated [24], as the potential for immune reactions related to allografts is minimized, and the biological and biomechanical properties are only partially affected [21,46]. Still, the grafts are not free of controversy, particularly regarding their association with the transmission of infectious agents. Some tissue processors incorporate methods that may markedly reduce this risk. It is critical to know your tissue bank provider to ensure their processing and preservation methods inactivate viruses but do not negatively alter the biomechanical and biochemical properties of the tissues intended for a particular clinical use [23].

Fresh-frozen and freeze-dried bone allografts induce more prompt graft vascularization, incorporation, and bone regeneration than fresh allograft [46]. Freeze drying produces a safer graft in terms of reducing the risk of immunologic responses in the donor and transmission of viral diseases. However, despite modern sterilization and storage methods, processing of allografts using freeze-drying techniques and treating the graft by hypotonic solutions, acetone, ethylene oxide, or gamma irradiation which can eliminate cellular and viral particles and therefore reduce the risk of infectious and transmissible diseases [45], the use of allografts is not completely safe [32,46]. These processes may destroy the bone cells and denature proteins present in the graft and alter osteoconductive and osteoinductive characteristics, essentially eliminating the osteogenic properties [24]. Therefore, freeze-dried allografts in comparison to autografts take longer to become revascularized and incorporated than autografts [21]. Freeze-drying procedure also reduces the mechanical strength of the graft, and the cost of processed and ready-to-use allografts is high [46,47]. The mineral component of the allogeneic bone can be removed by demineralization to obtain demineralized bone matrix (DBM) which has osteoinductive and partly osteoconductive properties [32]. DBM revascularizes quickly, and its biological activity is attributed to proteins and various growth factors present in the extracellular matrix [22]. Given these major disadvantages, allografts are not the perfect substitute for autograft.

### Xenografts

Another alternative to autogenous bone grafts are xenografts, also known as heterologous or xenogenic grafts [48]. Xenografts are harvested from one individual and transplanted into another individual of a different species. The common available xenografts are derived from coral (Biocoral^®^, natural coral; Biocoral Inc, Wilmington, New Castle, DE, USA), porcine, and bovine sources [48,49]. Xenogenous bone grafts are a theoretically unlimited supply of available material if they could be processed to be safe for transplantation in humans [48]. A major concern with bovine-derived products is the potential transmission of zoonotic diseases and prion infections such as bovine spongiform encephalitis (BSE) [17,49]. Xenografts, similar to allograft, lose their osteogenic and partly osteoinductive properties during the processing to counteract their antigenic properties and prevent transmission of infection. Xenografts produce poor clinical outcome [17]; however, new insights have been presented.

Several studies have been conducted to treat bony defects, non-unions, and pathologic bone fractures by application of different types of bone grafts (Table 3) [50-53]. In most of them, autologous bone grafts have been suggested as the gold standard, and other methods are compared with them [4,54], yielding variable levels of effectiveness when compared to autogenous bone grafts.

**Table 3:** Comparison of various bone grafts in several experimental and clinical studies

**Reference**	**Model of defect**	**Graft options**	**Model of study**	**Effects**
Emami et al. [50]	Radial bone defect	Iliac crest autograft and bone marrow plus the autograft	Experimental study in15 rabbits	Bone marrow plus the autograft caused high tolerance to maximum load and bending stiffness
Keskin et al. [11]	Ulnar bone defect	Autograft, bovine xenograft, and xenograft-autogenous bone marrow	Experimental study in 80 rabbits	Xenograft achieved the worst results. Combination of xenograft with autogenous bone marrow led to promising outcome
Pereira-Junior et al. [33]	Radial bone defect	Cancellous bone autograft vs. granular polyurethanes containing castor oil	Experimental study in 20 rabbits	Autograft showed higher and faster bone regeneration than castor oil-based polyurethane containing biocompatible and osteointegrative properties
Bigham et al. [3]	Radial bone defect	Fresh autogenous cortical bone vs. xenogenic bovine DBM	Experimental study in 20 rabbits	Fast healing without complications with xenogenic bovine DBM similar to autograft, but autograft group was superior to DBM only radiographically
Bigham et al. [51]	Radial bone defect	Xenogenic bovine DBM vs. xenogenic bovine fetal growth plate	Experimental study in 20 rabbits	With both grafting groups, healing was faster, despite the fetal growth plate which was radiographically superior to DBM
Shafiei et al. [14]	Radial bone defect	Fresh cortical autograft vs. fresh cortical allograft	Experimental study in 20 rabbits	Autograft was radiographically but not biomechanically and histopathologically superior to allograft
Athanasiou et al. [12]	Femoral condyle defect	Autogenous, allograft-DBM, bovine cancellous bone xenograft and calcium phosphate hydroxyapatite and calcium phosphate substitutes	Experimental study in 90 rabbits	The best results obtained with the use of autograft, followed by bovine xenografts, allograft, and ultimately, the other substitutes had similar results
Bansal et al. [4]	Tibial plateau fracture	Bovine cancellous xenograft	Clinical study, 19 patients	Obtained promising outcome, reduced operative time and bleeding good effects on bone healing
Putzier et al. [20]	Lumbar segmental spondylodesis	Autogenous vs. allogenic iliac crest cancellous bone graft	Clinical study, 40 patients	Both grafts attained equivalent fusion rate without implant complications and accordingly similar clinical outcome
Keles et al. [52]	Intraosseous periodontal defect	Combined autogenous cortical bone (ACB) and guided tissue regeneration (GTR) vs. ACB alone	Clinical study, 12 patients	Both the two groups resulted in improvement in clinical and radiological characteristics
Thuaksuban et al. [63]	Alveolar cleft defect	Autogenous bone alone vs. autogenous bone with deproteinized bovine bone (DBB)	Clinical study, 30 patients	Duration of hospital stay, the average operation time, intraoperative blood loss, and post-operative pain were less; recovery was faster in patients receiving DBB with autogenous cancellous bone graft
Faldini et al. [53]	Aseptic forearm non-union	Bone allograft with plate	Clinical study, 14 patients	High forearm alignment rate and improved forearm function led to bone healing
Scaglione et al. [6]	Long bone non-union	Autologous concentrated bone marrow-derived cells combined with dried bone allograft (DBM)	Clinical study, 19 patients	Complete healing in 15 patients (78.9%)

Keskin et al. [11] evaluated the effectiveness of autologous bone marrow on the healing of ulnar bone defects filled with bovine-derived xenografts in rabbits. The bony defect in the ulnae was produced by excising a 1-cm-long bone segment from the 3-cm proximal segment of the right distal radioulnar joint. The bone defects were treated simultaneously with bovine-derived xenograft, a combination of xenograft and bone marrow or, on the fifth day following the filling of the segment, with the xenograft and autogenous bone graft. They concluded that when xenografts were combined with autogenous red bone marrow, the drawbacks of xenografts were compensated; therefore, their incorporation into the recipient bed was significantly enhanced. In addition, they concluded that the spongy xenograft may provide a suitable medium for osteogenesis by bone marrow cells. Furthermore, some other studies have suggested that bone marrow injection could have more promising effects with no significant complication on bone healing in comparison with bone grafting [50,55].

Lubboc (Lubboc^®^; Osteocell SA, Athens, Greece) is a xenogenous-based purified trabecular bone matrix which mainly contains collagen type I and hydroxyapatite [12]. Athanasiou et al. [12] compared the histological properties of several widely used bone graft substitutes. For this purpose, they produced a 4.5-mm diameter hole in the lateral femoral condyle of both knees of 90 rabbits, allocated to six experimental groups. The bone defects were filled with various grafts including autograft, demineralized bone matrix crunch allograft (Grafton^®^; Osteotech, Inc., Eatontown, NJ, USA), bovine cancellous bone xenograft (Lubboc^®^), calcium phosphate hydroxyapatite substitute (Ceraform^®^; Teknimed, Vic-en-Bigorre, France), calcium sulfate substitute (Osteoset^®^; Synthes, West Chester, PA, USA), and no filling (control). The animals were euthanized at 1, 3, and 6 months after implantation, and the tissue samples from the implanted sites were histologically evaluated. The highest histological grades were obtained with the use of cancellous bone autograft. Bovine xenograft was the second best in the histological scale grading. The other substitutes were similar but inferior to both allograft and xenograft.

Recently, the effects of xenogenic bovine fetal DBM, commercial DBM, omentum, omentum-calf fetal DBM, cortical autograft, and xenogenic cartilage powder on the healing of tibial defects in a dog model has been investigated [56]. Overall, the omentum and omentum-DBM groups were superior to the control group but inferior to the autograft, commercial DBM, calf fetal DBM, and calf fetal cartilage groups.

Acellularization of soft and hard connective tissues such as tendons, ligaments, and bones reduces or even eliminates the immunogenicity associated with allografts and xenografts and, therefore, may be effective in enhancing incorporation of these grafts [57-60]. Multiple physical, chemical, and enzymatic methods have been used to remove cytoplasmic and nuclear antigens with preservation of the extracellular matrix structure and maintenance of mechanical and functional characteristics [58,60]. Ionic detergents such as sodium dodecyl sulfate (SDS) solubilize cell membranes and, given their tendency to denature proteins, also impair tissue structure. Using non-ionic detergents (such as Triton X) results in partial preservation of the structure of the acellularized tissue [57,60]. Zhang et al. [59] compared different methods such as NaCl + SDS, trypsin/EDTA, trypsin/EDTA + Triton X-100, Triton X-100, Triton X-100 + SDS, and freezing at -70°C followed by using Trypsin/EDTA + Triton X-100 to acellularize intrasynovial flexor tendons of rabbit. Among these agents, the best results regarding acellularization were obtained by freezing at -70°C followed by trypsin/EDTA + Triton X-100. Moreover, Elder et al. [57] evaluated the effects of various acellularization treatments on tissue-engineered articular cartilage constructs, including cellularity and biochemical and biomechanical properties as well as collagen content, using a two-phased approach after 4 weeks of culture. In the first phase, five treatment regimens were assessed, including 1% SDS, 2% SDS, 2% Triton X-100, 2% tributyl phosphate (TnBP), and hypotonic followed by hypertonic solution which were used for either 1 or 8 h, and then a 2-h wash in PBS. In phase II, the best treatment from phase I (2% SDS) was applied for 1, 2, 4, 6, or 8 h. Treatment with 2% SDS for 1 or 2 h significantly decreased the DNA content of the tissue while maintaining the biochemical and biomechanical properties. On the other hand, 2% SDS for 6 or 8 h led to complete histological acellularization, with complete elimination of cell nuclei, but substantial reduction of the compressive properties. Following this study, the treatment with 2% SDS for 1 or 2 h was the most effective and promising method for cartilage acellularization. Indeed, it resulted in complete acellularization while maintaining the physiological functional properties. Finally, Vavken et al. [58] compared the effectiveness of Triton X, trypsin, and SDS in acellularization of the porcine anterior cruciate ligament (ACL) and showed that Triton X is the most effective reagent for acellularization of the porcine ACL.

### Bone tissue engineering

Tissue engineering is the ‘final’ option in managing bone loss. Tissue engineering can involve the use of scaffolds, healing promotive factors (e.g., growth factors), and stem cells [17]. Tissue engineering is defined as ‘a process that affects the structure and architecture of any viable and non-viable tissue with the aim to increase the effectiveness of the construct in biologic environments’ [61]. Therefore, all the non-fresh grafts which are processed for acellularization belong to the tissue engineering category. In fact, acellularization is the basic tissue engineering technology described for allograft and xenografts [58]. This method of tissue engineering has been used for many years to decrease the antigenicity of the viable grafts [58,59]. Newer approaches have been developed, and newer tissue-engineered products have recently been introduced.

### Tissue scaffolds

Scaffolds are the most important issue in tissue engineering and could be divided into two main categories including biological (natural or organic) and synthetic (artificial) materials [5,22]. The former are natural polymers such as collagen type I or DBM [24,62,63]. Porous metals, bioactive glasses, synthetic polymers such as polylactic acid (PLA) and polyglycolic acid (PGA), and calcium phosphate ceramics such as hydroxyapatite (HA) and tricalcium phosphates (TCP) are examples of synthetic materials [2,24,27,32,64].

The traditional technologies used to acellularize the biologic grafts aiming to mimic characteristics of the autografts in the defect area started the basis of bone tissue engineering [58,59]. With this approach, the architecture of the graft was not altered, and the healing characteristics of such non-viable acellularized graft could not be increased [47]. Newer technologies used different materials to produce grafts, the architecture of which could be designed according to clinical needs. Synthetic materials are often selected as tissue engineering material in producing scaffolds because their polymeric molecules are commercially available and there is no need for special processing prior to use [65,66]. Using various tissue engineering technologies, different scaffolds, each with advantages and disadvantages, have been produced for bone tissue engineering applications (Table 4). In addition, scanning electron microscopy (SEM) images of several polymers have been provided in Figure 3.

**Table 4:** Advantages and disadvantages of some of the biologic and synthetic tissue-engineered polymers

**Tissue-engineered polymer**	**Advantages**	**Disadvantages**
Collagen	Major component of ECM, high availability, easy to purify from living organisms, non-antigenic, biodegradable, biocompatible and bioreabsorbable, non-toxic, biological plastic due to high tensile strength, formulated in a number of different forms	High cost of pure type I collagen, variability of isolated collagen, hydrophilicity leading to swelling and more rapid release, side effects such as bovine spongiform encephalopathy (BSF) and mineralization, low cell differentiation and inadequate ability to form bone
Chitosan	High biodegradability, biocompatibility, adsorption properties, ability to support cell differentiation, promotion of growth and differentiation of osteoblasts in cell culture, porous structure, flexible, good mechanical properties, and suitability for cell ingrowth	Not osteoconductive, inadequate bone formation ability, allergic reactions, and low solubility
Alginate	Easy to mix, manipulate, and use; non-toxic; biodegradable nature; less expensive; with quick setting time	Less accurate reproduction of detail, poor dimensional stability, messy to work with it, low mechanical stability (microparticles prepared only with calcium alginate)
Calcium phosphate	Excellent biocompatibility, bioactivity, optimal bone implant contact, easy preparation during surgery, minimal bone cavity, complete adaptation to the bone cavity, good setting *in situ*, excellent biological properties, potential resorbability, good molding capabilities, and easy manipulation	Low mechanical resistance, brittleness and low flexural/tensile strength

**Figure 3:** **SEM images.** Alginate **(A)**, alginate-chitosan **(B)**, chitosan **(C)**, chitosan-collagen **(D)**, mesenchymal stem cells cultured on the scaffold collagen (C)-dl-lactic acid-glycolic acid (PLGA) (P) medium **(E)**, and synthesized porous HA scaffold **(F)**. The scaffolds used for bone tissue engineering must be porous (scalebars **(A**-**D**, **F)** 100 μm, **(E)** 500 μm)*.*

To produce a scaffold, the biologic tissues should be degraded to their components and then redesigned according to the tissue engineering goals [67,68]. Such constructs are specific for one or two materials (e.g., collagen + hydroxyapatite, collagen + chitosan) and therefore have low antigenicity compared with cadaveric grafts [66,67]. Several characteristics have been suggested for the tissue-engineered constructs, including porosity, suitable pore size and shape, fiber alignment and orientation, fiber density, internal and external architecture, hydrophilicity, and hydrophobicity, including water uptake, binding, and delivery [65,69]. Regardless of the composition of the scaffolds, the abovementioned characteristics are crucial for their osteoconductive properties [34]. Since the materials should be substituted by the new bone, another important criterion is their resorbability. Degradation of the polymers is based on enzymatic or hydrolytic pathways [34,70]. Polymeric scaffolds have unique properties, such as biodegradation. Natural polymers are considered as the first biodegradable biomaterials, while synthetic biodegradable polymers can be produced under controlled conditions [34,71]. Bioactive ceramics, such as HA, TCP (TCP is more quickly biodegradable than HAP), and bioactive glasses, react with physiological fluids [71]. However, their biodegradability is often insufficient, limiting their potential clinical use. This issue can be overcome by blending synthetic and natural polymers or using composite materials that improve the scaffold properties such as biodegradability. These products are often named ‘hybrid’ [17,71-73].

In general, tissue-engineered constructs have low molecular density and high pore size, and their fiber alignment and size could vary based on the nature of the injury and the recipient tissue [74]. Scaffolds must be highly porous to allow cell ingrowth and facilitate neovascularization of the construct [71]. Average pore size, pore size distribution, pore volume, pore interconnectivity, and pore shape are important parameters to consider when designing a scaffold [74]. Pore size is very important: if the pores are too small, they will be occluded by the cells—this will prevent cellular penetration, extracellular matrix production, and neovascularization in the inner architecture of the scaffold. A pore size of 200–350 μm is optimal for bone ingrowth and facilitates osteoconduction [71].

### Natural-based materials used for tissue scaffolding

Natural- or biologic-based materials are taken from biologic-based tissues, and xenografts may be the best source for these later products. The advantages of natural-based scaffolds are that they have significantly superior biocompatibility, biodegradability, regenerative characteristics (e.g., osteoinduction, osteoconduction, osteogenesis, and osteointegration) than those of synthetic materials, but their immunological behavior is variable in different species and is also related to the type of application [75-79].

### Collagen

Collagens are among the most widely present in the human body, providing strength and structural stability to various tissues, from the skin to bone [78]. Collagen (collagen type I), the major organic component of ECM of the bone, is the most popular biologic materials used to produce biologically based tissue-engineered grafts (Table 4) [75,78,80]. Recent investigations tried to increase the biocompatibility, biodegradability, and regenerative capability of tissue-engineered-based scaffolds by incorporation of collagen into the structure of different composites. Surface modification of different bone scaffolds with collagen has been in the focus of many recent studies. Using aligned collagen fibers in the scaffold improved cellular proliferation, and differentiation to osteoblasts are obtained [78]. Collagen scaffolds have also been used as biomaterial carriers for bone morphogenetic proteins. Using a rat ectopic bone formation model, rhBMP-2 was injected into a collagen matrix and the results showed that using collagen, it is possible to functionally deliver bone-based growth factors to produce new bone formation *in vivo*[81]. Despite their excellent bioactivity, collagen-based scaffolds have low mechanical properties and are susceptible to substantial shrinkage during cell culture, which limits their potential applications in tissue engineering of bone. The effects of fish collagen peptides (FCP) on collagen synthesis, quality, and mineralization, using an osteoblastic MC3T3-E1 cell culture system, have been recently investigated: FCP exerts a positive effect on osteoblastic cells in terms of collagen synthesis, quality, and mineralization, thereby suggesting the potential utility of FCP for bone tissue engineering [82]. Moreover, a combination of collagen-chitosan-calcium phosphate microparticles has been produced which was then fused with glycolic acid. Incorporation of collagen into this bone graft substitute increases the biocompatibility and degradation profile of the composite [83].

### Chitosan

Chitosan, a linear polysaccharide with many commercial and biomedical uses due to its properties which allow it to rapidly clot blood, has recently gained approval in the USA and Europe for use in bandages and other hemostatic agents, quickly stopping bleeding and reducing blood loss, with a 100% survival of otherwise lethal arterial wounds in swine [84].The chitosan salts can be mixed with other materials (such as alginate) to make them more absorbent or to vary the rate of solubility and bioabsorbability of the chitosan salt. Chitosan salts are biocompatible and biodegradable making them useful as absorbable hemostats [85]. The chitosan salt may be placed on an absorbable backing. The absorbable backing may be synthetic (for instance, made from existing absorbable suture materials e.g., Tephaflex polymer; Tepha Medical Devices, Lexington, MA, USA) or natural (e.g., cellulose or gelled/solidified honey) [84]. The properties of chitosan also allow it to be used in transdermal drug delivery; it is mucoadhesive, reactive, can be produced in many different forms, and has a positive charge under acidic conditions. This molecule will maintain its structure in a neutral environment but will solubilize and degrade in an acidic environment. Hence, chitosan can be used to transport a drug to an acidic environment, where the chitosan packaging will then degrade, releasing the drug to the desired environment [85]. Given its unique properties, chitosan has been used in combination of various materials for bone tissue engineering purposes. Tridimensional composite scaffolds composed of chitosan and calcium phosphate have been developed and characterized. Air drying of this scaffold enhances its bioactivity. Given its optimum strength, degradation resistance, and cell-supportive characteristics, chitosan can be used for bone tissue engineering [86].

### Alginate

Alginic acid, also called algin or alginate, is an anionic polysaccharide distributed widely in the cell walls of brown algae where, binding with water, it forms a viscous gum. In extracted form, it quickly absorbs water, with a water absorption capacity of 200–300 times its own weight. It is sold in filamentous, granular, or powdered forms. A novel stem cell delivery system composed of collagen and alginate as the core and shell, respectively, has been developed. This fibrous carrier has been shown promising to enable the encapsulation of tissue cells and their delivery into damaged target tissues, including bone with defect tunability for bone tissue engineering [87].

### Elastin

Similar to collagen, elastin is a key structural protein found in the ECM of most tissues; yet, very little is known about the response of bone cells to elastin or its derivatives. Recently, a novel class of ECM-based composite scaffolds with collagen and a genetically engineered polymer, elastin-like polypeptide (ELP) has been designed and produced. By embedding the elastin within collagen scaffolds, it is possible to expect superior mechanical properties and drug release characteristics compared to collagen scaffolds alone. Elastin also enhances osteogenic differentiation of stem cells and regulates cells behavior *in vitro*[88].

### Cellulose

Cellulose is an organic compound and an important structural component of the primary cell wall of green plants, many forms of algae, and the oomycetes, and is secreted by some bacteria to form biofilms. Cellulose is the most abundant organic polymer on Earth [89]. Cellulose is used to make hydrophilic and highly absorbent sponges, beneficial in combination with other materials for bone tissue engineering applications [90]. A cellulose- and collagen-based micro-/nanostructured scaffold has been recently produced. After culturing human osteoblasts on the scaffold, the scaffold supported an optimum adhesion and phenotype maintenance of cultured cells as reflected by higher levels of osteogenic enzyme alkaline phosphatase and mineral deposition compared to control polyester micro-/nanostructured scaffolds of identical pore properties [90].

### Synthetic polymeric materials

Several *in vitro* and *in vivo* researches tried to optimize synthetic-based, tissue-engineered scaffolds in order to be useful in bone regenerative medicine. A single-walled carbon nanotube (SWCNT) and polylactic-*co*-glycolic acid (PLGA) composite has been developed recently. After seeding with human MSCs and osteoblasts, the composite imparted beneficial cellular growth capability and gene expression, and mineralization abilities were well established suggesting its potential application in bone regeneration [91]. As another strategy, a combination of different polymers has been tried to increase the cell cytocompatibility of the synthetic-based scaffolds. Poly(*l*-lactide) and poly(caprolactone triol) are some examples. Using such combination, new membranes promoted the rat osteoblastic cell behavior *in vitro* (e.g., migration, attachment, proliferation, and matrix production) [92]. Surface modification and coating is another strategy to enhance bioactivity of the synthetic scaffolds. Silica nanoparticles have been applied onto the fiber surface of an interbonded three-dimensional polycaprolactone (PCL) fibrous tissue scaffold. The nanoparticle layer was found to improve the fiber wettability and surface roughness. Thus, it enhanced osteoblast attachment, proliferation, and alkaline phosphatase activities [93]. Despite many beneficial characteristics of synthetic materials in bone healing and regeneration, their biocompatibility, biodegradability, and regenerative properties are still suboptimal compared to natural-based scaffolds. Therefore, many attempts have been made to combine synthetic with natural materials. Recently, poly(d,l-lactide-*co*-glycolide) has been combined with a naturally bioceramic hybrid material, nanonized pearl powder, as an osteoinductive material: the scaffold was able to influence osteoblast behavior *in vitro*[94]. The benefits associated with polyhydroxyalkanoates (PHA) in tissue engineering include high immunotolerance, low toxicity, and biodegradability. Poly(3-hydroxybutyrate-*co*-3-hydroxyhexanoate) (PHBHHx), a molecule from the PHA family of biopolymers, shares these features. Collagen has been used with PHA to increase the biocompatibility of the scaffold and to support cell proliferation and osteogenic differentiation *in vitro*[95].

There is an increasing demand for an injectable cell-coupled three-dimensional (3D) scaffold to be used as bone fracture augmentation material. To address this demand, a novel injectable osteogenic scaffold called PN-COL was developed, using cells, a natural polymer (collagen type I), and a synthetic polymer (PCL). The injectable nanofibrous PN-COL is produced by interspersing PCL nanofibers within pre-osteoblast cell embedded collagen type I. This simple yet novel and powerful approach provides a great benefit as an injectable bone scaffold over other non-living bone fracture stabilization polymers, such as polymethylmethacrylate and calcium content resin-based materials. The advantages of injectability and the biomimicry of collagen were coupled with the structural support of PCL nanofibers to create cell-encapsulated Injectable 3D bone scaffolds with intricate porous internal architecture and high osteoconductivity. The effects of PCL nanofiber inclusion within the cell-encapsulated collagen matrix have been evaluated for scaffold size retention and osteocompatibility, as well as for MC3T3-E1 cells osteogenic activity. At structural analysis, this novel bioactive material was chemically stable enough in an aqueous solution for extended periods without using crosslinking reagents, but it is also viscous enough to be injected through a syringe needle. Data from long-term *in vitro* proliferation and differentiation suggests that PN-COL scaffolds promote osteoblast proliferation, phenotype expression, and formation of mineralized matrix [96]. A novel dicalcium phosphate anhydrate/poly(lactic acid) (DCPA/PLA) composite nanofiber, which mimics the mineralized collagen fibrils via biomimetic *in situ* synthesis and electrospinning for hard tissue regenerative medicine, has been produced. Addition of poly(ethylene glycol), as a copolymer source, produced more stable and efficient electrospun jets and aided in the electrospun ability of the PLA nanofibers incorporating the nanocrystallites [97].

### Calcium phosphate and its derivatives

Different types of mono-, bi-, and tricalcium phosphate bioceramics and molecules have been extensively used in bone tissue engineering researches and developments [68]. Hydroxyapatite is a naturally occurring mineral form of calcium apatite. Up to 50% of the bone's weight is a modified form of hydroxyapatite (known as bone mineral). Carbonated calcium-deficient hydroxyapatite is the main mineral of which dental enamel and dentin are composed [98]. Hydroxyapatite crystals are also found in the small calcifications (within the pineal gland and other structures) known as corpora arenacea or ‘brain sand’. Both the calcium phosphate and apatite forms have wide applications in bone tissue engineering [99]. Several authors have used such materials alone or in combination with other materials such as collagen, alginate, and chitosan in order to develop new scaffolds and tissue engineering strategies [98-107].

Recently, a biomimetic and bioactive tissue-engineered bone construct (porous nanocrystalline hydroxyapatite (nHA)/chitosan scaffolds) via a cold atmospheric plasma (CAP) treatment for directed osteogenic differentiation of human bone marrow MSCs has been introduced [98]. A new hybrid material (CMC-HA) containing HA in a carboxymethylcellulose (CMC)-based hydrogel was developed. The strategy for inserting HA nanocrystals within the hydrogel matrix consists of making the freeze-dried hydrogel to swell in a solution containing HA microcrystals. When the composite CMC-HA hydrogel was characterized and seeded with osteoblasts MG63 line, the scaffold with HA enhanced cell proliferation and metabolic activity and promoted production of mineralized extracellular matrix more than that observed for the scaffold without HA [102]. Sagar et al. [108] evaluated the complete healing of critical size defect made in the proximal tibia of rabbits, using nanohydroxyapatite/gelatin and chemically carboxymethylated chitin (nHA/gel/CMC) scaffold construct. The architecture indices analyzed by microcomputed tomography showed a significant increase in the percentage of bone volume fraction, with reconciled cortico-trabecular bone formation at the sites treated with nHA/gel/CMC constructs compared to controls. At histology and fluorescence labeling, the uniformly interconnected porous surface of the scaffold construct enhanced osteoblastic activity and mineralization.

Collagen has been extensively used with HA and or TCP to produce bone scaffolds. A bone-inspired material has been recently obtained by incorporating collagen in the liquid phase of α-tricalcium phosphate cement, either in solubilized or in fibrilized form. This material was able to set *in situ*, giving rise to a calcium-deficient hydroxyapatite (CDHA)/collagen composite. The composite controls the cell behavior to accelerate and trigger osteogenic differentiation *in vitro*[99]. A collagen-hydroxyapatite (Col-HA) composite through controlled *in situ* mineralization on type I collagen fibrils with nanometer-sized apatite crystals was designed and produced. After culturing the scaffolds with MSCs, the porous Col-HA composites had good biocompatibility and biomimetic properties and supported bone regeneration and formation [101].

A combination of collagen and HA has been used *in vivo*. Recently, a biomimetic collagen-apatite scaffold composed of collagen fibers and poorly crystalline bone-like carbonated apatite nanoparticles was developed to improve bone repair and regeneration. *In vivo*, the scaffold enhanced new bone formation in mice [106]. In addition, the effect of resorbable collagen membranes on critical size defects in rabbit tibiae filled with biphasic calcium phosphate has been investigated: biphasic calcium phosphate functioned well as a scaffold and allowed mineralized tissue formation. Furthermore, the addition of absorbable collagen membranes enhanced bone gain compared with non-membrane-treated sites [109].

The application of porous HA-collagen as a bone scaffold represents a new trend of mimicking the specific bone extracellular matrix. Application of HA in reconstructive surgery has shown that it is slowly invaded by the host cells. Therefore, implant compatibility may be augmented by seeding cells before implantation. Human primary osteoblasts were seeded onto innovative collagen-gelatin-genipin (GP)-HAp scaffolds. *In vitro* attachment, proliferation, and colonization of human primary osteoblasts on collagen-GP-HAp scaffolds with different percentages of HA (10%, 20%, and 30%) all increased over time in culture, but comparing different percentages of HA, they seem to increase with decreasing of HA component [105]. A tricomponent osteogenic composite scaffold made of collagen (Coll), HA, and poly(*l*-lactide-*co*-*ϵ*-caprolactone) (PLCL) has been recently developed. This Coll/HA/PLCL composite scaffold was combined with human osteoblast-like cells. The composite is highly porous, enabling osteoblast-like cell adhesion and growth [100]. Jung et al. [110] elucidated the role of collagen membranes (CMs) when used in conjunction with bovine hydroxyapatite particles incorporated with collagen matrix (BHC) for lateral onlay grafts in dogs. This strategy leads to superior new bone formation and bone quality compared with bone graft alone.

Calcium phosphate ceramics, specifically β-tricalcium phosphate (β-TCP) and synthetic HA, have recently been used in composites and in fibrous composites formed using the electrospinning technique for bone tissue engineering applications. Calcium phosphate ceramics are sought because they can be bone bioactive, so that apatite forms on their surface, facilitates bonding to bone tissue, and is osteoconductive [103]. In a recent study, the bioactivity of electrospun composites containing calcium phosphates and their corresponding osteogenic activity was investigated. Electrospun composites consisting of (20/80) HA/TCP nanoceramics and poly(*ϵ*-caprolactone) were fabricated, and the results demonstrated that after seeding the hybrid scaffold with human MSCs, the cells not only showed greater osteogenic differentiation but also proliferated and produced more bony matrix *in vitro*[103].

The combination of TCP and HA is another strategy. Bone healing and biodegradation patterns of three types of Ca-P ceramic particles with various HA/β-TCP weight ratios (pure β-TCP, biphasic Ca-P (BCP) with a HA/β-TCP weight ratio of 60/40 (BCP 60/40), and BCP with an HA/β-TCP weight ratio of 20/80 (BCP 20/80)) were investigated [106]. Four 8-mm-diameter defects were produced in ten rabbits. Three of the defects in each rabbit were separately and randomly filled with one of the three experimental Ca-P ceramic particles, and the fourth was filled with blood clots (control). After 2 and 8 weeks, BCP 60/40 and BCP 20/80 exhibited a similar bone healing and biodegradation patterns with regard to both individual particles and the total augmented area *in vivo*.

Piccinini et al. [111] implanted a new mineralogical formulation, HA/tetracalcium phosphate (TTCP), as a biomaterial for bone regeneration in the maxillary sinus of rats. After 17 weeks from implantation, HA/TTCP synthetic bone graft performed very well as osteoconductive material: bone graft contact was found very high, and bone volume and vital bone showed an ideal bone density for implant placement. Farahpour et al. [112] radiographically evaluated the effects of biphasic calcium phosphate scaffold with 5%, 10%, and 20% of porosity on cortical bone repair in rabbits. They showed that TCP + HA scaffold is an osteoconductive and osteoinductive biomaterial. TCP + HA scaffold can increase the amount of newly formed bone and more rapid regeneration of bone defects. Velasquez et al. [104] reported the *in vitro* and *in vivo* behavior of α-tricalcium phosphate (α-TCP) and also α-TCP with either 1.5 or 3.0 wt.% of dicalcium silicate (C2 S). The *in vivo* behavior of the ceramics matched the *in vitro* results, independent of the C2 S content in α-TCP. A fully mineralized new bone growing in direct contact with the implants was found under the *in vivo* conditions. The bioactivity and biocompatibility of the implants increased with the C2 S content in α-TCP. The C2 S-doped ceramics also favored a phase transformation of α-TCP into CHA, which is important for full implant integration during the natural bone healing processes.

The hybrid rapid prototyping (RP) scaffold of PLGA/β-TCP skeleton with collagen I/apatite sponge composite coating is a promising candidate for bone tissue engineering. The osteogenic potential of synthetic β-tricalcium phosphate in a hydroxyl sulfate matrix (β-TCP/HS) and human DBM putty has been investigated in rabbits [113]. In each animal, two bone defects (8-mm length × 3-mm width × 3-mm depth) were produced in the left and right regions of the mandible, respectively. The defect on one side was filled with β-TCP/HS (group A) or DBM putty (group B), while the defect on the opposite side was left unfilled to serve as a control site. After 1 to 6 weeks, β-TCP/HS and human DBM putty showed osteogenic activity and supported new bone formation.

### Bioactive glass

Several variations of glass beads called Bioglass (US Biomaterials, Alachua, FL, USA) are currently being developed, and one formulation (PerioGlas) has been approved in the USA for periodontal use. The beads are composed of silica (45%), calcium oxide (24.5%), disodium oxide (24.5%), and pyrophosphate (6%). When implanted, they bind to collagen, growth factors, and fibrin to form a porous matrix to allow infiltration of osteogenic cells [114]. Recently, a novel nanocomposite hydrogel made of collagen and mesoporous bioactive glass nanoparticles with surface amination has been developed [115]. The addition of bioglass into the collagen hydrogel significantly increases the bioactivity of the scaffold and improves its mechanical properties; this novel strategy would therefore be suitable for bone tissue engineering applications [115]. Moreover, the bioactive glass foam produced by sol–gel is an osteoinductive material with a network of interconnected macropores necessary for cell colonization. It has been shown that bioactive glass can differentiate human adipose-derived stem cells into osteoblasts, *in vitro*[116]. Moreover, Gu et al. [117] used scaffolds composed of a mixture of two different bioactive glasses (silicate 13–93 and borate 13-93B3) to evaluate their response to osteogenic MLO-A5 cells *in vitro* and their capacity to regenerate bone in rat calvarial defects *in vivo*. The scaffolds can guide bone regeneration and have a controllable degradation rate. A combination of glass and HA has also been used in bone regeneration. Fredericks et al. [118] determined the performance characteristics of a novel silicate-substituted HA bone graft substitute (BGS), SiCa-P EP (Baxter Healthcare/ApaTech, Elstree, UK), in a stand-alone mode, a stand-alone with bone marrow aspirate (BMA) mode, and an extender mode with iliac crest autograft (ICBG) in a rabbit posterolateral spine fusion model. The SiCa-P EP utilized as a stand-alone, as a stand-alone with BMA, and as an autograft (ICBG) extender produced results that were clinically and radiographically similar to ICBG.

### Healing promotive factors

Healing promotive factors such as growth factors have been extensively used to treat bony defects and for osteoinduction. Some growth factors such as vascular endothelial growth factor (VEGF), TGF-β, PDGF, and BMPs such as BMP-2, BMP-7, and IGF are present in the healthy bone matrix and are expressed during bone healing [32,34,119]. These factors can regulate vascularization and induce proliferation and differentiation of the osteoblasts and their precursors, so they can be useful in improving the healing processes [32].

Bone morphogenetic protein-2 (BMP-2) is a potent osteoinductive cytokine that plays a critical role during bone regeneration and repair. In the extracellular environment, sulfated polysaccharides anchored covalently to glycoproteins such as syndecan and also non-covalently to fibronectin fibers have been shown to bind to BMP-2 through a heparin-binding domain and regulate its bioactivity [37]. The supramolecular peptide amphiphile nanofibers, which integrate the biological role of syndecan and fibronectin, have been controlled and designed to form as a network within the pores of an absorbable collagen scaffold. The hybrid biomaterial enhanced significantly bone regeneration in a rat critical size femoral defect model using BMP-2 in amounts that are one order of magnitude lower than that required for healing in this animal model. Presence of more mature bone in the new ossified tissue was noted when a low dose of BMP-2 was delivered using the biomimetic supramolecular system [80]. Cha et al. [120] determined the efficacy of BMP-2 in a BHC carrier to augment bone formation in a canine nasal sinus model. Following preparation of bilateral sinus access windows, BHC alone (control) or loaded with *Escherichia coli*-derived BMP-2 at 0.1 mg/mL was implanted in four animals, and BHC loaded with *E. coli*-derived BMP-2 at 0.5 and 1.5 mg/mL was implanted in four animals. The animals were euthanized at 20 weeks. Histometric analysis showed significantly enhanced bone formation for the BMP-2 groups compared with control. BMP-2 in a BHC carrier, even at the low 0.1-mg/mL concentration, induced osteogenic activity, thus enhanced the local bone formation in a canine sinus model. Jang et al. [121] determined whether a HA/β-TCP ratio of 20/80 impregnated with rhBMP-2 enhances new bone formation in rat calvarial defect model. rhBMP-2 significantly induced new bone formation. In addition, Stancoven et al. [122] evaluated the potential of rhBMP-2 soak-loaded on to an absorbable collagen sponge (ACS) to induce local bone formation compared with the clinical reference DBM and to investigate potential additive/synergistic effects of exogenous parathyroid hormone (PTH). Critical size (8 mm) through-through calvaria osteotomy defects in 160 adult male rats were randomized to receive one of the eight interventions: rhBMP-2/ACS, DBM, ACS, or serve as controls (empty defects) combined or not with systemic PTH. Four to eight weeks post-surgery, rhBMP-2/ACS significantly stimulated local bone formation, whereas bone formation was significantly limited in the DBM group. Systemic application of PTH provided no discernible additive/synergistic effects on local bone formation. Liu et al. [123] produced a novel biomimetic bone scaffold composed of calcium sulfate hemihydrate (CSH), collagen, and nanohydroxyapatite (nHAC). rhBMP-2 was introduced into CSH/nHAC. The scaffolds with or without rhBMP-2 were implanted into a critical size defect model in the femoral condyle of rabbit. The results of plain radiography, micro-CT, and histological observation indicated that more new bone was formed in rhBMP-2 group.

Although many reports confirmed the beneficial effects of BMP on bone regeneration and quality, some others showed their ineffectiveness on regeneration of non-weight bearing bone healing. In an investigation, the biomechanical properties of calvarial bone regenerated with derivations of a commercially available rhBMP-2-based system were evaluated. Standardized calvarial defects were produced in 23 adult male canines. These defects were treated with rhBMP-2 on one of the several carriers. After 24 weeks, the biomechanical properties of the rhBMP-2-generated bone were compared to those of the controls with a modified punch-out test. They concluded that rhBMP-2-generated calvarial bone is significantly less protective against trauma than native bone at 6 months.

Hsu et al. [124] evaluated a combination therapy (TrioMatrix^®^; Pioneer Surgical, Inc., Marquette, MI, USA) composed of DBM, hydroxyapatite, and a nanofiber-based collagen scaffold in a rodent spine fusion model. Thirty-six athymic rats that underwent a posterolateral intertransverse spinal fusion were randomly assigned to one of the five treatment groups: ACS alone (negative control), 10 μg rhBMP-2 on ACS (positive control), TrioMatrix^®^ (Osteotech, Inc., Eatontown, NJ, USA), Grafton^®^, and DBX^®^ (Synthes Inc.). Both TrioMatrix^®^- and rhBMP-2-treated animals demonstrated 100% fusion rates as graded by manual palpation scores 8 weeks after implantation. This rate was significantly greater than those of the ACS, Grafton^®^, and DBX^®^ groups. Notably, the use of TrioMatrix^®^ quantified by micro-CT led to a greater fusion mass volume when compared to all other groups, including the rhBMP-2 group. T2-weighted axial MRI images of the fusion bed demonstrated a significant host response associated with a large fluid collection with the use of rhBMP-2; this response was significantly reduced with the use of TrioMatrix^®^. In another study, BMP-7 or DBM was implanted in a rabbit tibial distraction model, and healing was compared to a non-treated control group. Neither of the treatments showed a changed healing pattern. Densities as measured by CT scan were not increased, and the only significant finding was an increased area of bone formation in the DBM-treated group (65% increase). These experimental results do not show an effect of these substances in this model of bone lengthening [125].

Combination of zoledronate and BMP-7 has also been tested *in vivo* to optimize bone healing. Zoledronic acid (INN) or zoledronate (marketed by Novartis (Basel, Switzerland) under the trade names Zometa, Zomera, Aclasta, and Reclast) is a bisphosphonate given intravenously. Zometa is used to prevent skeletal fractures in patients with cancers such as multiple myeloma and prostate cancer, as well as for treating osteoporosis. It can also be used to treat hypercalcemia of malignancy and can be helpful for treating pain from bone metastases and fractures [126]. Yaman et al. [127] examined the effects of systemic zoledronic acid administration on the osseointegration of HA-coated and resorbable blast material surface (RBM) implants in a rabbit tibial model. Histomorphometric analyses showed significant improvement in the osseointegration of implants in the RBM-surface zoledronic acid group compared with the HA-coated zoledronic acid group. The results suggest that systemic zoledronic acid administration may improve osseointegration of titanium implants in bone. In rats, Mathavan et al. [128] investigated the role of combination of allograft + BMP-7 + systemic zoledronate (ZA) on bone healing and regeneration. Femoral osteotomies were performed on 82 male Sprague Dawley rats and fixed with intramedullary Kirschner wires. The rats were randomized into seven groups: (i) saline, (ii) autograft, (iii) allograft, (iv) allograft + BMP-7, (v) autograft + ZA, (vi) allograft + ZA, and (vii) allograft + BMP-7 + ZA. The rats were euthanized at 6 weeks. Complete radiological healing was seen in all rats in the BMP-7 groups. The callus volume was larger, and the calluses were denser with allograft + BMP-7 + ZA than in all other groups. Mechanical testing yielded a substantially higher peak force with the allograft + BMP-7 + ZA combination than all other groups, with a 59% increase in the peak force observed in the osteotomized femurs of the allograft + BMP-7 + ZA group compared to the control femurs, whereas significant decreases of 22%–27% were observed in the saline or bone-graft alone groups. Allograft combined with the anabolic effect of BMP-7 and the anti-catabolic effect of zoledronate is more efficient than autograft alone.

TGF-β1 is crucial in the development, induction, and repair of bone. The effect of local application of a graft DBM along with TGF-β1 in a model of open osteotomy induced experimentally in dogs has been investigated [129]. An open osteotomy of the tibia was produced in young male dogs. On the fifth week, there was an improvement and restoration of bone architecture in animals treated with a graft containing TGF-β1 (5 ng/mL) compared with the control and graft groups, as evidenced by early formation of wide callus and bone regeneration. In addition, local application of TGF-β1 led to an increase in collagen and proteolytic activity. More immunopositive osteoclast and mesenchymal cells were found in the bone tissue from animals treated with TGF-β1 compared with the control group. Ozturk et al. [130] investigated the role of a novel hydroxyapatite containing gelatin scaffold with and without local vascular endothelial growth factor as the synthetic graft material in the treatment of critical-sized tibial bone defects in rabbits. After 6 weeks, the administration of VEGF on the graft exerted a positive effect in the early phases of fracture healing but had no effect after 12 weeks.

Alendronic acid or alendronate sodium, sold as Fosamax by Merck (Whitehouse Station, NJ, USA), is a bisphosphonate drug for osteoporosis and several other bone diseases. It is marketed alone as well as in combination with vitamin D. On February 6, 2008, the US FDA approved the first generic versions of alendronate, which were marketed by Barr Pharmaceuticals (Montvale, NJ, USA) and Teva Pharmaceuticals (Horsham Road North Wales, PA, USA) [131]. Mathijssen et al. [132] investigated the role of several materials and drugs on bone healing. Twenty-five goats received eight bone conduction chambers in the cortical bone of the proximal medial tibia. Five concentrations of alendronate (0, 0.5, 1, 2, and 10 mg/mL) were tested in combination with allograft bone and supplemented with cefazolin (200 μg/mL). Allograft not supplemented with alendronate and cefazolin served as control. In addition, allograft mixed with DBM, with and without alendronate, was tested. After 12 weeks, a dose–response relationship for local application of alendronate was detected. Local application of cefazolin had no effect on bone remodeling.

Simvastatin is considered a stimulator of bone formation. However, the half-life for simvastatin is generally 2 h, therefore not likely to be biologically active *in vivo*. To overcome this limitation, Jiang et al. [133] created a system to slowly release simvastatin *in vitro* and *in vivo*. They constructed a polylactic-*co*-glycolic acid/hydroxyapatite nanofibrous scaffold to carry simvastatin and implanted the construct into calvaria bone defect models. After 4 to 8 weeks post-implantation, they indicated that polylactic-*co*-glycolic acid/hydroxyapatite/simvastatin scaffold induced bone formation more efficiently than controls.

Platelet-rich plasma (PRP) is a simple way of delivering growth factors [134,135]. The combination of human PRP with HA may be a promising alternative for reconstruction and regeneration of critical size defects in animal models [134,136]. More recently, a combination of PRP with silicon stabilized HA/TCP scaffold has been effective in rabbit calvarial defect (Skelite™; Millenium Biologix Corporation, Kingston, Ontario, Canada). Using such strategy, significant osteoid-like matrix and new bone deposition together with higher cellularity, more abundant osteoid deposition, and more regular collagen fibers could be seen in micro-CT and histologic analysis when compared to scaffold alone. Moreover, *in vitro* migration assays confirmed the chemotactic effect of PRP to endothelial and osteoprogenitor cells. Addition of PRP influenced the local tissue microenvironment by providing key cryptic factors for regeneration, thereby enhancing the progenitor cell recruitment and collagen and bone matrix deposition and creating a bridging interface between the scaffold and bone [137]. Some controversies exist in the effectiveness of PRP. The effect of autologous PRP on the early phases of osteoinduction by allogenic DBM in rabbit intramuscular positions has shown that addition of PRP to DBM had a negative effect on the early phases of osteoinduction at 3 weeks [138]. Faratzis et al. [139] investigated the effect of autologous PRP on the osteogenic potential of a biphasic synthetic graft material composed of HA/β-TCP in critical size cranial defects in rabbits. Autologous PRP in addition to a biphasic HA/β-TCP synthetic graft material had no effect on bone healing after 2, 4, and 6 weeks of implantation.

In another study, bone regeneration in three groups of rat calvaria treated with DBM from the Iranian Tissue Bank Research and Preparation Center (Tehran, Iran), DBM from Hans Biomed Corporation (Seongdong, Seoul, Korea), and or leaving the cavity empty were studied [140], using albumin as carrier. Bone regeneration after 1, 4, and 8 weeks of implantation was evaluated. The two types of DBM had a significant difference in bone regeneration. This difference was attributed to the type of carriers. Albumin could improve mineralization and bioactivity compared with control carriers.

### Stem cells

The combination of stem cells with scaffolds as a polytherapy is a new option. Collagen and demineralized bone powder have been used to produce a novel scaffolds for bone tissue engineering. Human periosteum-derived cells (PD cells) were cultured on this scaffold: the hybrid scaffolds exhibited greater osteoinductive potential than collagen scaffolds. The PD cells with hybrid scaffolds possessed higher ALP activity, calcium deposition, and superior behavior (e.g., attachment, differentiation, and proliferation) than those with collagen scaffolds [141].

The feasibility of applying calcined bovine bone (CBB) coated with allograft bone marrow mesenchymal stem cell (BMSC)-sheet as a 3D scaffold material in bone healing has been investigated recently. The new scaffold material was implanted into osteoporosis rat cranial bone defects and critical size bone defects (8-mm diameter). The CBB-BMSC-sheet combination had a stronger potential in osteogenic differentiation and mineralized formation both *in vitro* and *in vivo* than CBB-BMSC combination. Three-dimensional reconstruction of micro-CT, H&E staining, and bone strength results showed that the area and volume of the newly formed bone in CBB-BMSC-sheet group was significantly higher than that of the CBB-BMSC group after 4 to 12 weeks [142].

Adipose-derived stem cells (ASCs) with multilineage differentiation capacities have been demonstrated as an alternative cell candidate for *in vitro* and *in vivo* bone regeneration. This suggests that they may be a potential candidate to repair the bone defects. Yang et al. [143] attempted to demonstrate the use of new biomimetic constructions of undifferentiated rabbit ASCs with fully interconnected porous β-TCP scaffolds encapsulated by collagen I hydrogel in the regeneration of a critical-sized defect of rabbit radii. Critical-sized defects in the left radii of rabbits were prepared and inserted with rASCs/collagen I/β-TCP scaffold composites or collagen I/β-TCP scaffold composites. Twelve weeks after implantation, the defects were almost completely repaired as confirmed by the presence of the cortical bone and medullary cavity. In addition, a greater number of ASCs in the scaffold enhanced osteogenesis in critical-sized defects. Pourebrahim et al. [144] compared bone regeneration of tissue-engineered bone from ASCs and autogenous bone graft in a canine maxillary alveolar cleft model. The undifferentiated cells were incubated with a HA/β-TCP scaffold in specific osteogenic medium for 21 days. Four mongrel dogs were prepared by removal of two of the three incisors bilaterally and a 15-mm defect in bone was created from the crest to the nasal floor. After healing, repair was followed by a tissue-engineered bone graft from ADCs on one side and cortico-cancellous tibial autograft on the other side. Bone regeneration was evaluated by histomorphometry on days 15 and 60 after implantation. The bone formation on the autograft sides was higher than on the stem cell sides at 15 and 60 days, and 45% and 96% versus 5% and 70%, respectively.

Pang et al. [145] observed the therapeutic effects of hybrid RP scaffolds comprising PLGA, β-TCP, collagen I, and apatite (PLGA/β-TCP-collagen I/apatite) on segmental bone defects in conjunction with combined bone marrow MSCs. The bone defect remained unconnected in the original RP scaffolds (PLGA/β-TCP) during the study. In hybrid RP scaffold group, woven bone united the radial defect at 12 weeks and consecutively remodeled into lamellar bone at 24 weeks post-operation and finally matured into cortical bone with normal marrow cavity after another 12 weeks. No bone formation but connective tissue was detected in the RP scaffold at the same time. Xuan et al. [146] produced polycaprolactone/HA tissue scaffolds with individualized grooves to repair the sternal defect. The defects were surgically produced in a sternocostal joint of Beagle dogs. The animals were allocated to one of the three groups (*n* = 6): no treatment group, PCL/HA group, and PCL/HA/BMSCs group. The application of the PCL/HA scaffolds with specific grooves resulted in satisfactory repair of the sternal defect. Furthermore, the BMSCs-seeded scaffolds enhanced the amount of bone ingrowth and seemed to be more promising. Calcium phosphate nanoparticles such as HA/fluorapatite (FA), with chitosan gel filled with unrestricted somatic stem cells (USSCs), have been used for healing calvarial bone in a rat model [147]. The combination of scaffold especially with USSC could be considered a useful method for bone regeneration.

In another study, autogenic and allogenic bone-marrow-derived MSCs were compared for repair of bone gap defect in rabbits. The defects were filled with HA alone, HA with autogeneic BM-MSCs, and HA with allogenic BM-MSCs. Histologically, increased osteogenesis, early and better reorganization of cancellous bone, and more bone marrow formation were discernible in treatment groups as compared to the control group. *In vitro* culture expanded allogenic and autogenic BM-MSCs induced similar but faster and better healing as compared to control [148].

### The newest approach in tissue engineering: three-dimensional printing

Three-dimensional printing (3DP) is a rapid prototyping technique that can create complex 3D structures by inkjet printing of a liquid binder onto powder biomaterials for tissue engineering scaffolds. Direct fabrication of scaffolds from 3DP, however, imposes a limitation on material choices by manufacturing processes. Novel additive manufacturing processes are increasingly recognized as ideal techniques to produce 3D biodegradable structures with optimal pore size and spatial distribution, providing adequate mechanical support for tissue regeneration while shaping ingrowing tissues [149]. With regard to the mechanical and biological performances of 3D scaffolds, pore size and geometry play a crucial role. Domingos et al. [150] used a novel integrated automated system for production and *in vitro* culture of 3D constructs, known as BioCell printing, to manufacture poly(*ϵ*-caprolactone) scaffolds for tissue engineering. The results clearly demonstrated the potential of the BioCell printing process to produce 3D scaffolds with reproducible well-organized architectures and tailored mechanical properties. More recently, Billiet et al. [151] reported on the combined efforts of material chemistry, engineering, and biology as a systemic approach for the fabrication of high-viability 3D-printed macroporous gelatin methacrylamide constructs. Lee et al. [152] reported an indirect 3DP approach wherein a positive replica of desired shapes was printed, using gelatin particles, and the final scaffold was directly produced from the printed mold. To produce patient-specific scaffolds that match precisely a patient's external contours, the authors integrated their indirect 3DP technique with imaging technologies and successfully produced custom scaffolds mimicking human mandibular condyle using polycaprolactone and chitosan for potential osteochondral tissue engineering. To test the ability of the technique to precisely control the internal morphology of the scaffolds, they produced orthogonal interconnected channels within the scaffolds using computer-aided-design models. Because very few biomaterials are truly osteoinductive, they modified inert 3D printed materials with bioactive apatite coating. The feasibility of these scaffolds to support cell growth was investigated using bone marrow stromal cells (BMSC). The BMSCs showed good viability in the scaffolds, and the apatite coating further enhanced cellular spreading and proliferation. This technique may be valuable for complex scaffold fabrication.

The ability to three-dimensionally interweave biological tissue with functional electronics could enable the creation of the bionic organs possessing enhanced functionalities over their human counterparts. Mannoor et al. [153] presented a novel strategy to overcome these difficulties via additive manufacturing of biological cells with structural and nanoparticle-derived electronic elements. As a proof of concept, they generated a bionic ear via 3D printing of a cell-seeded hydrogel matrix in the anatomic geometry of a human ear, along with an intertwined conducting polymer consisting of infused silver nanoparticles. This allowed for *in vitro* culturing of cartilage tissue around an inductive coil antenna in the ear, which subsequently enables readout of inductively coupled signals from cochlea-shaped electrodes. The printed ear exhibited enhanced auditory sensing for radio frequency reception, and complementary left and right ears could listen to stereo audio music. Overall, their approach suggests a means to intricately merge biologic and nanoelectronic functionalities via 3D printing.

### Gene therapy

Gene therapy consists of transfer of genetic information to the target cells and may introduce a safe and effective strategy to induce bone healing. Gene therapy can be used for delivery of growth factors in tissue engineering [1,2]. The vehicle for gene delivery can be either viral (adenovirus, retrovirus, and adeno-associated virus) or non-viral (liposomes) [22,154]. However, this approach has a series of limitations, including trans-infection of the target cells with the foreign genes [1,154]. Furthermore, an unresolved issue of gene therapy is to target the right gene at the right location in the right cells and express it for sufficiently long at the right time, while minimizing adverse reactions [155]. A short controlled expression is desirable and often sufficient to accelerate bone healing, while achieving permanent or long-term expression of a therapeutic gene is more difficult. Therefore, providing controlled and sufficient expression by adaptation of gene therapy to tissue engineering is a key and critical aspect in this field [61,156].

### Commercial bone graft substitutes

The ideal bone-graft substitute is biocompatible, biodegradable, osteoconductive, osteoinductive, structurally similar to bone, easy to use, and cost-effective. Within these parameters, a growing number of bone graft alternatives are commercially available for orthopedic applications, including reconstruction of cavitary bone deficiency and augmentation in situations of segmental bone loss and spine fusion. They are variable in their composition and their claimed mechanisms of action [70]. Based on the FDA and American Academy of Orthopedic Surgeons' reports and the manufacturers' information, many bone graft substitutes have been approved for clinical use. This large variability and options make it hard to select a graft when reconstruction of an injured bone is a purpose. A summary of commercially available bone graft substitutes has been provided in Tables 5, 6, 7 and 8.

**Table 5:** Commercially available bone graft substitutes: part 1

**Company**	**Commercially available product**	**Composition**	**Commercially available forms**	**Claimed mechanisms of action**	**Level of evidence**	**FDA status**
AlloSource	AlloFuse™	Heat-sensitive copolymer with DBM	Injectable gel and putty	Osteoconduction	Case reports	510(k) cleared
				Biodegradable	Animal studies	
				Osteoinduction	Cell culture	
Biomet Osteobiologics	ProOsteon^®^ 500R	Coralline-derived hydroxyapatite/calcium carbonate (HA/CC) composite	Granular or block	Osteoconduction	Human studies	510(k) cleared
				Biodegradable	Case reports	
					Animal studies	
	InterGro^®^	DBM in a lecithin carrier	Paste, putty, and mix with HA/CC composite granules	Osteoconduction	Case reports	510(k) cleared
				Biodegradable	Animal studies	
				Osteoinduction	Every lot tested for osteoinduction	
	BonePlast^®^	Calcium sulfate with or without HA/CC composite granules	Various volumes of powder and setting solution	Osteoconduction	Case reports	510(k) cleared
				Biodegradable	Animal studies	
DePuy Spine	HEALOS^®^ Bone Graft Replacement	Mineralized collagen matrix	Variety of strip sizes	Osteoconduction	Peer-reviewed, published human studies	510(k) cleared
				Creeping substitution	Case reports	
				Osteoinduction	Animal studies	
				Osteogenesis when mixed with bone marrow aspirate		
	CONDUIT^®^ TCP Granules	100% β-TCP	Granules	Osteoconduction	Case reports	510(k) cleared
				Biodegradable	Animal studies	
Exactech	Opteform^®^	DBM and cortical cancellous chips suspended in gelatin carrier	Formable putty or dry powder ready to be hydrated with autologous diluents or saline	Osteoconduction	Human studies	510(k) cleared
				Biodegradable	Case reports	
				Osteoinduction	Animal studies	
				Osteogenesis when mixed with autogenous bone graft	Every lot tested *in vivo* for osteoinduction	
	Optefil^®^	DBM suspended in gelatin carrier	Injectable bone paste; dry powder ready to be hydrated with blood or saline	Osteoconduction	Human studies	510(k) cleared
				Biodegradable	Case reports	
				Osteoinduction	Animal studies	
				Osteogenesis when mixed with autogenous bone graft	Every lot tested *in vivo* for osteoinduction	
	Optecure^®^	DBM suspended in a hydrogel carrier	Dry mix kit delivered with or buffered saline mix with patient's autogenous bone graft or autologous diluents	Osteoconduction	Human studies	510(k) cleared
				Biodegradable	Case reports	
				Osteoinduction	Animal studies	
				Osteogenesis when mixed with autogenous bone graft	Every lot tested *in vivo* for osteoinduction	
	Optecure^®^ + CCC	DBM and CCC suspended in a hydrogel carrier	Dry mix kit delivered with buffered saline or mix with patient's autogenous bone graft or autologous diluents	Osteoconduction	Animal studies	510(k) cleared
				Biodegradable	Every lot tested *in vivo* for osteoinduction	
				Osteoinduction		
				Osteogenesis when mixed with autogenous bone graft		
	OpteMx™	HA/TCP biphasic combination	Granules, sticks, rounded wedges, wedges, and cylinders in several sizes	Osteoconduction	Human studies	510(k) cleared
				Biodegradable	Case reports	
				Compressive strength of 400 psi	Animal studies	
				Osteogenesis and limited osteoinduction when mixed with bone marrow aspirate		

Data were extracted based on the reports of FDA, American Academy of Orthopedic Surgeons, and information provided by the manufacturers.

**Table 6:** Commercially available bone graft substitutes: part 2

**Company**	**Commercially available product**	**Composition**	**Commercially available forms**	**Claimed mechanisms of action**	**Level of evidence**	**FDA status**
Integra Orthobiologics/(IsoTis OrthoBiologics)	Accell 100™	DBM putty	Injectable putty	Osteoconduction	Human studies	510(k) cleared
				Bioresorbable	Case reports	
				Osteoinduction	Animal studies	
					Every DBM lot tested for osteoinduction	
	Accell Connexus^®^	DBM plus reverse phase medium	Injectable putty	Osteoconduction	Human studies	510(k) cleared
				Bioresorbable	Case reports	
				Osteoinduction	Animal studies	
					Every DBM lot tested for osteoinduction	
	Accell TBM™	Total bone matrix, 100% preformed	Various-sized strips	Osteoconduction	Human studies	510(k) cleared
				Bioresorbable	Case reports	
				Osteoinduction	Animal studies	
					Every DBM lot tested for osteoinduction	
	Integra Mozaik™	80% highly purified B-TCP	Strip and putty	Osteoconduction	Animal studies	510(k) cleared
		20% highly purified type-1 collagen		Bioresorbable	Case reports	
LifeNet Health	Optium DBM^®^	DBM combined with glycerol carrier	Formable putty (bone fibers) and injectable gel (bone particles)	Osteoconduction	Human studies	510(k) cleared
				Bioresorbable	Case reports	
				Osteoinduction	Animal studies	
	IC Graft Chamber^®^	DBM particles and cancellous chips	Lyophilized and packaged in various sizes within a delivery chamber	Osteoconduction	Animal studies	Regulated under CFR 1270 and 1271 as a human tissue and 510(k) cleared
				Bioresorbable	Case reports	
				Osteoinduction		
				Designed to be used with blood, PRP, or bone marrow to enhance DBM activity		
	Cellect DBM^®^	DBM fibers and cancellous chips	Provided in a specialized cartridge	Osteoconduction	Animal studies	Regulated under CFR 1270 and 1271 as a human tissue and 510(k) cleared
				Bioresorbable	Case reports	
				Osteoinduction		
				Designed for the retention of osteoprogenitor cells		
Medtronic Spinal & Biologics	INFUSE^®^ Bone Graft	rhBMP-2 protein on an absorbable collagen sponge	Multiple kit sizes	Bioresorbable carrier	Human studies (level I and level III data)	PMA approved for fusion with spinal cage
				Osteoinduction	Case reports	PMA approved for open tibia fractures with IM nail
				Chemotaxis of stem cells; indirect osteogenesis	Animal studies	
	MasterGraft^®^ Granules	Biphasic calcium phosphate	Granules	Osteoconduction	Animal studies	510(k) cleared
				Bioresorbable		
	MasterGraft^®^ Matrix	Calcium phosphate and collagen	Compression resistant block	Osteoconduction	Animal studies	510(k) cleared
				Bioresorbable		
	MasterGraft^®^ Putty	Calcium phosphate and collagen	Moldable putty	Osteoconduction	Animal studies	510(k) cleared
				Bioresorbable		

Data were extracted based on the reports of FDA, American Academy of Orthopedic Surgeons, and information provided by the manufacturers.

**Table 7:** Commercially available bone graft substitutes: part 3

**Company**	**Commercially available product**	**Composition**	**Commercially available forms**	**Claimed mechanisms of action**	**Level of evidence**	**FDA status**
Medtronic Spinal & Biologics	Progenix™ DBM Putty	DBM in type1 bovine collagen and sodium alginate	Ready to use injectable putty	Osteoconduction	Animal studies	510(k) cleared
				Bioresorbable		
				Osteoinduction		
	Osteofil^®^ DBM	DBM in porcine gelatin	Injectable paste and moldable strips	Osteoconduction	Animal studies	510(k) cleared
				Bioresorbable	Case reports	
				Osteoinduction		
MTF/Synthes	DBX^®^	DBM in sodium hyaluronate carrier	Paste, putty mix, and strip	Osteoconduction	Human studies	510(k) cleared
				Bioresorbable	Case reports	
				Osteoinduction	Animal studies	
NovaBone/ MTF	NovaBone^®^	Bioactive silicate	Particulate and putty	Osteoconduction	Case reports	510(k) cleared
				Bioresorbable	Animal studies	
				Osteostimulation		
Orthovita	Vitoss^®^	100% β-TCP and 80% β-TCP/20% collagen	Putty, strip, flow, morsels, and shapes	Osteoconduction	Published human studies	510(k) cleared
				Bioresorbable	Case reports	
					Animal studies	
Osteotech	Grafton^®^	DBM combined with glycerol	Formable putty, injectable gel, putty mixed with chips, flexible sheets, and matrix	Osteoconduction	Published human studies	510(k) cleared
				Bioresorbable	Case reports	
				Osteoinduction	Animal studies	
	Graft on Plus^®^	DBM combined with a starch carrier	Paste	Osteoconduction	Case reports	510(k) cleared
				Bioresorbable	Animal studies	
				Osteoinduction		
Regeneration Technologies	BioSet™	DBM combined with natural gelatin carrier	Injectable paste, injectable putty, strips, and blocks with cortical cancellous chips	Osteoconduction	Human studies	510(k) cleared
				Bioresorbable	Case reports	
				Osteoinduction	Animal studies	
					Every lot tested *in vivo* for osteoinduction	
Smith & Nephew	VIAGRAF	DBM combined with glycerol	Putty, paste, gel, crunch, and flex	Osteoconduction	Animal studies	510(k) cleared
				Bioresorbable		
				Osteoinduction		
Stryker Biotech	OP-1^®^ Implant	rhBMP-7 with type 1 bone collagen	Lyophilized powder reconstituted to form wet sand	Bioresorbable scaffold	Human studies (level I data)	HDE approval for long bone non-unions
				Osteoinduction	Case reports	
					Animal studies	
	OP-1^®^ Putty	rhBMP-7 with type 1 bone collagen	Lyophilized powder reconstituted to form putty	Bioresorbable scaffold	Human studies (level I data)	HDE approval for revision posterolateral fusion
				Osteoinduction	Case reports	
					Animal studies	
	Calstrux™	Tricalcium phosphate with carboxymethylcellulose	Moldable putty	Osteoconduction	Animal studies	510(k) cleared
				Bioresorbable		

Data were extracted based on the reports of FDA, American Academy of Orthopedic Surgeons, and information provided by the manufacturers.

**Table 8:** Commercially available bone graft substitutes: part 4

**Company**	**Commercially available product**	**Composition**	**Commercially available forms**	**Claimed mechanisms of action**	**Level of evidence**	**FDA status**
Synthes	Norian^®^ SRS^®^ Fast Set Putty	Calcium phosphate	Moldable putty	Osteoconduction	Human studies	510(k) cleared
				Bioresorbable	Case reports	
					Animal studies	
	chronOS^®^	β-tricalcium phosphate	Granules, blocks, and wedges	Osteoconduction	Animal studies	510(k) cleared
				Bioresorbable		
	Calceon^®^ 6	Calcium sulfate	Pellets	Osteoconduction	Animal studies	510(k) cleared
				Bioresorbable		
	OSTEOSET^®^	Surgical grade calcium sulfate	Various sized pellets	Osteoconduction	Human studies	510(k) cleared
				Bioresorbable	Case reports	
					Animal studies	
Wright Medical Technology	MIIG^®^ X3	High strength surgical grade calcium sulfate	Minimally invasive injectable graft for compression fractures	Osteoconduction	Human studies	510(k) cleared
				Bioresorbable	Case reports	
					Animal studies	
	CELLPLEX^®^	Tricalcium phosphate	Various sized granules	Osteoconduction	Case reports	510(k) cleared
				Bioresorbable	Animal studies	
	ALLOMATRIX^®^	DBM with/without CBM in surgical grade calcium sulfate powder	Various volumes of injectable/ formable putty	Osteoconduction	Human studies	510(k) cleared
				Bioresorbable	Case reports	
				Osteoinduction	Animal studies	
					Cell culture	
	ALLOMATRIX^®^ RCS	DBM with CACIPLEXTM Technology in surgical grade calcium sulfate powder	Various volumes of formable putty	Osteoconduction	Animal studies	510(k) cleared
				Bioresorbable		
				Osteoinduction		
	IGNITE^®^	DBM in surgical grade calcium sulfate powder to be mixed with bone marrow aspirate	Percutaneous graft for problem fractures	Osteoconduction	Human studies	510(k) cleared
				Bioresorbable	Case reports	
				Osteoinduction	Animal studies	
					Cell culture	
Zimmer	CopiOs^®^ Bone Void Filler	Dibasic calcium phosphate and Type I collagen	Sponge and paste	Osteoconduction	Case reports	510(k) cleared
				Bioresorbable	Animal studies	
				Osteogenesis and osteoinduction when mixed with bone marrow aspirate		
	CopiOs^®^ Cancellous Bone Graft	Bovine bone	Cancellous chips, cancellous cubes and wedges	Osteoconduction	Case reports	510(k) cleared
					Animal studies	
	Puros^®^ Demineralized Bone Matrix	DBM putty	Putty	Osteoconduction	Every lot tested *in vivo* for osteoinduction	100% derived from allograft tissue
				Bioresorbable		FDA clearance not required
				Osteoinduction		

Data were extracted based on the reports of FDA, American Academy of Orthopedic Surgeons, and information provided by the manufacturers.

Based on the data provided in Tables 5, 6, 7 and 8, most of the bone graft substitutes have been licensed under FDA 510(k) program, but some of them have been regulated under CFR 1270 and 1271 programs in addition to 510(k). Manufacturers of AlloSource, Biomet Osteobiologics, DePuy Spine, Exactech, Integra Orthobiologics/(IsoTis OrthoBiologics), LifeNet Health, Medtronic Spinal & Biologics, MTF/Synthes, NovaBone/MTF, Orthovita, Osteotech, Regeneration Technologies, Smith & Nephew, Stryker Biotech, Synthes, Wright Medical Technology, and Zimmer are some examples of companies that have produced several commercially available bone graft substitutes applicable in clinical practice.

Despite many advances in tissue engineering technologies, most of the commercially available bone graft substitutes are natural-based materials that have been used and processed with the cadaver allograft and xenograft origins.

Regarding the available products, DBM, the most popular option, has been extensively produced and is available on market. DBM has both osteoconduction and osteoinduction and is biodegradable, making it an ideal graft substitute. It is available as injectable paste and putty, graft, gel, crunch, and flex and often is conjugated or embedded with collagen type I, alginate, gelatin, sodium hyaluronate, glycerol, starch, and calcium sulfate. Regardless of the DBM carrier, the material can also be mixed with bone marrow aspirate prior to surgery. The second well-known option is the calcium phosphate group including mono-, bi- and tricalcium phosphate. They are often available in conjugation with collagen type I and carboxymethylcellulose, and all of them are osteoconductive and biodegradable products as injectable paste, moldable putty, and various-sized pellets. rhBMP-2 and rhBMP-7 proteins on an absorbable collagen sponge are other biodegradable options with some osteoinductive characteristics. Commercial bovine bone matrix, allograft bone matrix, calcium sulfate, and bioactive silicate are other available options with variable osteoconductivity and osteoinductivity.

## Discussion

To design and produce an efficient bone graft, the researchers and orthopedic surgeons should have sufficient knowledge of the characteristics of grafts such as osteogenesis, osteoinductivity, and osteoconductivity, and their other advantages and disadvantages. Autografts are the gold standard for bone regeneration. Among the available strategies to improve fracture healing and enhance the outcome of incorporation of the grafts, tissue engineering is a suitable option [9,10,17]. An ideal tissue-engineered product should have characteristics similar to those of autografts without their limitations [17].

The bone scaffolds should additionally be highly porous and have pores of suitable sizes at all locations of the scaffold to provide an optimal environment for new bone matrix and bone regeneration [17]. Furthermore, growth factors such as basic fibroblastic growth factor [74,157,158] which may affect cell functions, proliferation, or differentiation; healing promotive agents such as hPRP [15,35,136]; and also *Tarantula cubensis* extract [134,159] can be included in the scaffolds to enhance the healing performance of the injured connective tissues. Agents such as glycosaminoglycans, including hyaluronic acid, chondroitin, and dermatan sulfate have modulatory roles in bone and fracture healing and can improve the quality of the tissue-engineered scaffolds [17,159]. More recently, zoledronate, simvastatin, and alendronate have been shown to have promising effects on bone healing and regeneration [128,132,133].

The vascularity of the scaffold is critical because if not present, the scaffold will undergo ischemia and the cells will die. Therefore, application of growth factors such as VEGF, PDGF, and FGF can be useful to stimulate angiogenesis in the scaffolds and the grafts [32,34]. A combination of stem cells with scaffolds and healing promotive factors, especially the growth factors, could be one possible strategy providing all the necessary characteristics for bone repair and regeneration.

None of the applied grafts has all the desirable characteristics such as biological safety, low donor morbidity, no size restriction, long shelf life, efficient cost and osteogenic, osteoinductive, osteoconductive, and angiogenic properties. Tissue engineering attempts to provide most or all of these features [18,69]. Tissue engineering is also able to induce repair and reconstruction of bone defects [17]. Combining the fundamentals of orthopedic surgery with knowledge from various sciences such as engineering, biology, chemistry, physics, and materials science can overcome the limitations of current therapies [9]. Advances in tissue engineering and biomaterials will provide more suitable tools to promote the migration, proliferation, and differentiation of bone cells and enhance bone fracture healing. Several problems remain that limit wide utilization of such options, including regulatory requirements, high costs, lack of randomized controlled human and animal studies, uncertain long-term results, and method-specific limitations. Although the literature contains a large number of studies on the effects of various agents on bone healing, it still is unclear which the best option is. Nevertheless, autograft remains the gold standard of grafting [12,20].

The near future of bone healing and regeneration is closely related to advances in tissue engineering. Perhaps polytherapy by using scaffolds, healing promotive factors, and stem cells together with the new advances in three- and four-dimensional printing of tissue-engineered constructs would be able to solve the current limitations in managing bone injuries.

## Conclusion

Bone grafting is one of the most commonly used options to treat large bone defects. Autografts remain the gold standard. Allografts, xenografts, and tissue-engineered-based grafts all have shortcomings. New strategies such as gene therapy, polytherapy by using scaffolds, healing promotive factors and stem cells, and finally three-dimensional printing are in their preliminary stages but may offer new exciting alternatives in the near future.

## Competing interests

The authors declare that they have no competing interests.

## Authors’ contributions

All authors had equal contribution in all parts of the study. AO, SA, AM, and NM designed the study and participated in data collection, manuscript preparation, and revision. All authors read and approved the final manuscript.
